RETRACTED

# Analysis of the Correlation between the Distribution of MTHFR Gene and the Severity and Renal Function of Elderly Patients with H-Type Hypertension

**DOI:** 10.1155/2022/8352005

**Published:** 2022-04-12

**Authors:** Chi Zhang, Zhijie Dou, Cui Zhao, Jun Li, Qiuping Xin, Yumei Feng, Yunbo Xie, Junjie Cao

**Affiliations:** Affiliated Hospital of Chengde Medical College, Chengde 067000, China

## Abstract

In order to investigate the correlation between the distribution of methylenetetrahydrofolate reductase (MTHFR, MR) C677T gene and the severity of disease and renal function in elderly patients with H-type hypertension, a total of 170 patients with H-type hypertension admitted to our hospital from September 2020 to February 2021 and 173 elderly patients with non-H-type hypertension during the same period are selected as the research objects and are respectively included in the observation group and control group. Baseline data and distribution of MR C677T genotype are compared between the two groups, influencing factors of H-type hypertension are analyzed by logistic regression analysis, and differences and correlation of homocysteine (Hcy) and estimated glomerular filtration rate (eGFR) levels in different MR C677T genotypes are compared. The influence of MR C677T genotype on the severity and renal function of patients with H-type hypertension is further analyzed. There are many influencing factors for H-type hypertension, including advanced age, high-sodium diet, and MR TT genotype. Patients with hypertension with these risk factors should be monitored. H-type hypertension has a high frequency of carrying TT genotype and T allele, and the TT genotype in H-type hypertension will affect the Hcy and eGFR levels. Therefore, Hcy level of H-type hypertension patients with TT genotype should be actively controlled to help control the disease and reduce kidney damage. MR TT genotype can be used as a reference index in the early screening of H-type hypertension.

## 1. Introduction

Hypertension is a common type of cardiovascular diseases, which can cause damage to the brain, kidney, heart, and other important organs. H-type hypertension refers to the abnormal increase of homocysteine (Hcy) in patients with hypertension. In China, H-type hypertension accounts for more than 70.00% of hypertension [1, 2]. Abnormal increase of Hcy will cause kidney damage and decrease of renal function, which will aggravate the condition of Hcy increase in patients with H-type hypertension, thus forming a vicious circle and posing a serious threat to the life and health of patients [3]. Methylenetetrahydrofolate reductase (MR) participates in and plays an important role in the decomposition and metabolism of Hcy. It has been pointed out that MR C677T gene has obvious genetic polymorphism in Chinese population, and the mutation of MR gene locus may be related to changes in Hcy metabolism and levels. Therefore, clarifying the distribution of MR C677T genotype in patients with H-type hypertension and its relationship with patients' condition and renal function has certain guiding value for early disease screening and diagnosis [4]. This study aims to study the distribution of MR C677T genotype in patients with H-type hypertension and its correlation with changes in Hcy and renal function so as to provide data support for improving the accuracy of early screening in patients with H-type hypertension by using C677T genotype and actively providing effective intervention measures.

RETRACTED

A total of 170 patients with H-type hypertension who visited our hospital from September 2020 to February 2021 are selected and assigned to the observation group, and 173 non-H-type elderly hypertension patients are included in the control group during the same period. The average age of the observation group is (58.87 ± 9.44) years, the male to female ratio is 78/92, the course of disease is (12.87 ± 5.29) years, and the ratio of technical secondary school or below to college or above is 80/90. The control group is 46∼78 years old, with an average of (56.77 ± 10.01) years old, and the male to female ratio is 85/88 cases. The disease duration is 2∼34 years, with an average of (12.62 ± 5.20) years. The ratio of technical secondary school or below to college or above is 84/89 cases. Inclusion criteria of the observation group: (1) H-type hypertension is diagnosed with Hcy ≥10 umol/L according to the diagnostic criteria of Chinese H-type hypertension expert consensus on diagnosis and treatment in 2016 [5]; (2) unconscious disorders and communication disorders can actively cooperate with research and examination and other operations [6–8]; (3) not in menstruation, pregnancy, and lactation [9, 10]; (4) clear research content and sign informed consent voluntarily [11, 12]; and (5) age ≥45. Exclusion criteria are as follows: (1) secondary hypertension [13, 14]; (2) systemic blood diseases, infectious diseases, and immune system diseases [15, 16]; (3) surgical treatment or blood transfusion within 3 months before the study [17, 18]; (4) suffering from malignant tumor [19, 20]; and (5) those who took vitamin B12, vitamin B6, folic acid, or other substances that affected serum Hcy level in the last 3 months [21]. It is consistent with the inclusion criteria (2)∼(5) of the observation group. This study has been approved by the medical ethics committee of our hospital.

RETRACTED

## 2. Detection Method

Subjects in the study are abstained from high-protein, high-fat, and high-sugar foods 3 days before blood collection and had a light diet. They are also fasting 12 hours before blood collection, and 5 ml of venous blood of the fasting external elbow is collected in the morning of the next day. After anticoagulation, the blood is stored in the refrigerator at −80°C. Genomic DNA of peripheral anticoagulant blood is extracted and primers are designed for MR C677T genotype. Primer sequence design and genotype detection are completed in the central laboratory of our hospital. A 25 *μ*L reaction system is prepared by 8.5 *μ*L H_2_O, 3.0 *μ*L template DNA, 2.5 *μ*L PCR mastermix 1, and 0.5 *μ*L primers, respectively. The reaction is repenetrated at 95°C for 5 min, and the denaturation lasted for 60 seconds at the same temperature. Annealing reaction is carried out at 59°C for 60 seconds, extension reaction is carried out at 72°C for 60 seconds, 36 cycles, and extension reaction is carried out at 72°C for 5 minutes. A 32 *μ*L restriction endonuclease reaction system is prepared with 2 *μ*l HINIendonuclease, 18 *μ*l dd H_2_O, 2 *μ*l 10 × Buffer R, and 10 *μ*l PCR products. The endonuclease reaction is digested overnight at 37°C. The endonuclease reaction is terminated by electrophoresis and stained with silver nitrate. After 35 min of staining, the genotypes such as CC type (wild type), CT type (heterozygous type), and TT type (mutant type) are determined by using an ultraviolet gel imager.

After fasting for 12h, 4 ml venous blood is collected in fasting state in the next morning, and centrifugation is performed at 3000 r/min rotation speed and 7 cm radius for 19 min. Serum is separated, and the plasma Hcy level is detected by ELISA (ELISA kit provided by Beijing Jiuqiang Biotechnology Co., Ltd.). Type DG 022A ELISA is used.

Estimated glomerular filtration rate (eGFR) is calculated using the modified Chinese formula C-AGFR4. For males, the formula is eGFR = (140 − age) × body weight (kg)/(0.818 × creatinine (*μ*mol/L)), female calculation formula: eGFR = (140 − age) × body weight (kg) /(0.818 × creatinine (*μ*mol/L)) × 0.85.

Statistical analysis is performed using the SPSS 24.0 software. The normally distributed measurement data are expressed as ($\bar{x}\pm s$), and the *t*-test is used; the multigroup data is expressed by the *F* test; the count data percentage *n* (%) is expressed, and the *x*^*2*^ test is used. Multivariate logistic regression analysis of the influencing factors of H-type hypertension. The correlation of MR C677T genotype with renal function, and Hcy level is analyzed by multiple linear regression.

## 3. The Clinical Results

### 3.1. Univariate Analysis of Differences in Clinical Baseline Data

The proportion of H-type hypertension patients aged ≥75 years and high-sodium diet significantly increased; the data are statistically different (*P* < 0.05).  Table 1 is univariate analysis of differences in clinical baseline data.

RETRACTED

### 3.2. Comparison of MR C677T Genotype and Distribution of Alleles C and T

The proportion of CC type and CT type genotype and the frequency of C allele are lower in the observation group, while the proportion of TT type genotype and the frequency of T allele in the observation group are higher, and the data are statistically different. *P* < 0.05, as shown in Table 2.

### 3.3. Risk Factors of H-type Hypertension Are Analyzed by Multivariate Logistic Regression

The factors (*P* < 0.05) are substituted as independent variables into the multifactor logistic regression model group of H-type hypertension for analysis, and the variable assignment values are shown in Table 3. The results show that age ≥75 years, high-sodium diet, and TT genotype are independent risk factors for H-type hypertension, as shown in Table 4.

### 3.4. Comparison of Hcy Levels among Different MR C677T Genotypes

The Hcy level in the TT genotype significantly increased than that in the CT genotype and CC genotype, and the Hcy level in the CT genotype significantly increased than that in the CC genotype, with statistical significance (*P* < 0.05).  Table 5 displays comparison of the Hcy gap of different MR C677T genotypes.

### 3.5. Comparison of Renal Function Level Differences among Different MR C677T Genotypes

EGFR level in the TT genotype significantly decreased than that in the CT genotype and CC genotype, and eGFR level in the CT genotype significantly decreased than that in CC genotype, with statistical significance (*P* < 0.05).  Table 6 presents comparison of differences in renal function levels among different MR C677T genotypes.

### 3.6. Multiple Linear Regression Analysis of the Correlation between MR C677T Genotype and Hcy and eGFR

With Hcy and eGFR as continuous variables and MR C677T genotype as independent variables, multiple linear regression analysis showed that TT genotype is positively correlated with Hcy and negatively correlated with eGFR.  Table 7 illustrates correlation of MR C677T genotype with Hcy and eGFR by multiple linear regression analysis.

## 4. Experimental Result Analysis

Hypertension patients under the effects of high pressure, high perfusion, and high filtration will cause functional impairment of renal artery and glomerulus, resulting in reduced renal function. Therefore, active control of hypertension is of great significance to prevent renal function injury. Hcy is a sulfur-containing amino acid, mainly produced by the human methionine metabolism, its oxidation process could damage the body organs and tissues of free oxygen, kidney function decline and kidney damage can lead to Hcy metabolic pathways blocked Hcy accumulation in great quantities, and this can lead to H-type hypertension.

RETRACTED

The occurrence of H-type hypertension is affected by a variety of factors, and previous studies have shown that diet and living habits will affect the level of Hcy, thus affecting the risk of H-type hypertension. Zhang et al. believed that advanced age is an independent risk factor for increasing the risk of H-type hypertension. In this study, age ≥75 years old and high-sodium diet accounted for a higher proportion in the observation group, and the two variables are independent risk factors for the occurrence of H-type hypertension, suggesting that people with age ≥75 years old and high-sodium diet and other risk factors are more prone to abnormal elevation of Hcy and H-type hypertension, which should be the focus of prevention. The effect of age and a high-sodium diet were analysed, and the causes of high blood pressure may be after age and the body's metabolism. It makes the renal function, metabolism of Hcy, and other nutrient absorption abilities to reduce, and a high-sodium diet will lead to patients unable to absorb enough folic acid and B vitamins. Thus, methionine circulation disorder is caused, which affects the effective utilization of Hcy and leads to a large accumulation of Hcy, thus causing H-type hypertension. Therefore, Hcy level should be regularly monitored for elderly patients with hypertension, and the occurrence of H-type hypertension should be actively prevented through rational planning of dietary and nutritional intake.

From the perspective of biogenetics, gene locus mutation can reduce the enzyme activity, and then inhibit the decomposition and metabolism of Hcy, and increase the level of Hcy accordingly. MTHFR gene contains 11 exons, which are located on chromosome 1 with a total length of about 17 KB, and the most common mutation site is nucleotide C-T site 677. Comprehensive analysis of MR C677T genotype distribution results and Hcy levels of different genotypes in H-type hypertension patients in this study showed that the TT genotype and T allele carrying frequency in H-type hypertension patients in the observation group are significantly higher than those in non-H-type elderly hypertension patients. Hcy levels in H-type hypertension patients with TT genotype are significantly higher than those in patients with CT and CC genotype, while the Hcy level of CT genotype is higher than that of the CC genotype. TT genotype is positively correlated with Hcy level. Dong Li et al. believed that patients with TT genotype had a significantly higher risk of developing H-type hypertension than those with CT and CC genotypes, which is consistent with the results of this study. It is further speculated that TT genotype and T allele might be the reasons for the occurrence of H-type hypertension and the aggravation of H-type hypertension caused by the increase of Hcy level. The mechanism may be that thymine (T) replaced cytosine (C) when the gene at C677 of MTHFR is mutated, resulting in the conversion of the coding codon of the gene to valine, resulting in the decrease of MTHFR enzyme activity. The enzyme activity of CT and TT genotype mutations is 65% and 30% of CC genotype, respectively, which leads to significant obstruction of Hcy methylation metabolism in the body, and thus Hcy cannot be removed from the body in a timely and effective manner, ultimately leading to abnormal increase in Hcy concentration and aggravation of H-type hypertension.

RETRACTED

Combined with the analysis of changes in renal function index (eGFR) in this study, eGFR level of patients with TT genotype is significantly lower than that of patients with CT and CC genotype, and eGFR level of CC genotype is the highest. TT genotype is negatively correlated with eGFR level, indicating that MR C677T gene polymorphism is related to reduced renal function. Jiao Fetyan et al. believed that high Hcy and MR C677T gene mutation is one of the main mechanisms of early renal damage. Analysis of its mechanism is as follows: The TT type mutation of MR C677T gene leads to abnormal increase of Hcy, and the high level of Hcy inhibits the transport of L-arginine cells in endothelial cells, resulting in low expression of nitric oxide synthase (NOS), which reduces the production of NO to a certain extent. Oxidative stress and inflammatory response are aggravated, leading to kidney damage and renal dysfunction. Therefore, H-type hypertension patients with MR C677T gene mutation will cause high Hcy levels and aggravate kidney damage. Effective measures should be taken to reduce the Hcy level in these patients, to play a positive role in preventing kidney injury, renal dysfunction, and controlling the progression of H-type hypertension.

## 5. Conclusion

Insufficient sample size and incomplete inclusion of reference variables still exist in this study, which limits the further analysis of this paper to some extent. It is necessary to add other factors that may affect H-type hypertension and other genotypes in subsequent studies. The paper further analyzes the correlation and mechanism of genetic and clinical factors with changes of Hcy and renal function indexes in H-type hypertension patients.

RETRACTED

Advanced age, high-sodium diet, and MR TT genotype are all risk factors for inducing H-type hypertension, and it is necessary to focus on the care of hypertensive patients with these risk factors. H-type hypertension patients have a higher frequency of TT genotype and T allele, and TT genotype is related to Hcy and eGFR levels of H-type hypertension patients. Hcy level of patients with active TT genotype control should be improved to control the disease and reduce kidney damage, and MR TT genotype can be used as a reference index for early screening of H-type hypertension.

## Figures and Tables

**Table 1:** Univariate analysis of differences in clinical baseline data.

Factors	Observation group (*n* = 170)	Control group (*n* = 173)	*x* ^*2*^	*P* value
Age (age)			13.210	<0.001
＜75	63 (37.06)	98 (56.65)		
≥75	107 (62.94)	70 (43.35)		

Sex			0.363	0.547
Male	78 (45.88)	85 (49.13)		
Female	92 (54.12)	88 (50.87)		

High-sodium diet			7.572	0.006
Yes	89 (52.35)	65 (37.57)		
No	81 (47.65)	108 (62.43)		

Degree of education			0.077	0.782
Technical secondary school and below	80 (47.06)	84 (48.55)		
College degree or above	90 (52.94)	89 (51.45)		

Physical exercise			0.071	0.790
Yes	86 (50.59)	90 (52.02)		
No	84 (49.41)	83 (47.98)		

Long-term mental tension			0.069	0.793
Yes	88 (51.76)	92 (53.18)		
No	82 (48.24)	81 (46.82)		

**Table 2:** Comparison of MR C677T genotype and distribution of alleles C and T.

Group	MR C677T genotype			MR C677T allele	
	CC	CT	TT	C	T
Observation group (*n* = 170)	30 (17.65)	60 (35.29)	80 (47.06)	120 (35.29)	220 (64.71)
Control group (*n* = 173)	87 (50.29)	54 (31.21)	32 (18.50)	228 (65.90)	118 (34.10)

*x* ^*2*^	40.649			375.125	
*P* value	<0.001			<0.001	

**Table 3:** Variable assignment table.

Factor	Variable	Assignment
Age (age)	*X*1	＜60 = 1, ≥75 = 2
High-sodium diet	*X*2	No = 1, Yes = 2
The MR C677T genotype	*X*3	CC = 1, CT = 2, TT = 3
High blood pressure type H	*Y*	No = 1, Yes = 2

**Table 4:** Multivariate logistic regression analysis of risk factors for H-type hypertension.

Property	*β*	S. E	Wald	*P* value	OR	95% CI	
						Lower limit	Top limit
Constant term	−4.1133	1.0125	16.5041	<0.001	—	—	—
Age ≥75 years	2.0564	0.4805	18.3154	<0.001	7.818	3.048	20.050
High-sodium diet	2.0454	0.4425	22.3132	<0.001	6.811	3.021	20.047
TT genotype	1.3823	0.2186	39.9703	<0.001	3.984	2.595	6.115

**Table 5:** Comparison of the Hcy gap of different MR C677T genotypes.

Genotype	Hcy (*μ*mol/L)
CC mould (*n* = 30)	10.25 ± 2.04
CT mould (*n* = 60)	16.56 ± 3.11^*∗*^
TT mould (*n* = 80)	20.46 ± 5.05^∗#^
*F*	2.543
*P* value	0.012

^*∗*^Compared with CC genotype <0.05; ^#^Compared with CT genotype <0.05.

RETRACTED

**Table 6:** Comparison of differences in renal function levels among different MR C677T genotypes.

Genotype	EGFR (mL/(min 1.73 m^2^))
CC mould (*n* = 30)	97.25 ± 32.24
CT mould (*n* = 60)	83.56 ± 26.13^*∗*^
TT mould (*n* = 80)	75.46 ± 21.22^∗#^
*F*	2.786
*P* value	0.005

^*∗*^Compared with CC genotype <0.05; ^#^Compared with CT genotype <0.05.

**Table 7:** Correlation of MR C677T genotype with Hcy and eGFR by multiple linear regression analysis.

Property	Hcy				EGFR			
	Β	S. E	*P* value	OR (95% CI)	*β*	S. E	*P* value	OR (95% CI)
CC mould	1.000	—	—	—	—	—	—	—
CT mould	0.015	0.031	0.558	0.945 (0.832∼1.043)	−0.018	0.023	0.343	0.842 (0.749∼1.052)
TT mould	0.189	0.014	0.017	1.842 (1.256∼3.483)	−0.134	0.016	0.012	1.789 (1.544∼3.558)

## Data Availability

The simulation experiment data used to support the findings of this study are available from the corresponding author upon request.
